# Influence of Weather Conditions on the Intercity Travel Mode Choice: A Case of Xi'an

**DOI:** 10.1155/2021/9969322

**Published:** 2021-08-23

**Authors:** Xiaowei Li, Qiangqiang Ma, Wenbo Wang, Baojie Wang

**Affiliations:** ^1^School of Civil Engineering, Xi'an University of Architecture & Technology, Xi'an 710055, China; ^2^CCCC First Highway Consultants Co. Ltd, Xi'an 710075, China; ^3^School of Transportation Engineering, Chang'an University, Xi'an 710054, China

## Abstract

To explore the influence of weather conditions on the choice of the intercity travel mode of travelers, four modes of traveler transportation were studied in Xi'an, China, in March 2019: airplane, high-speed rail, conventional train, and express bus. The individual characteristics of travelers and intercity travel activity data were obtained, and they were matched with the weather characteristics at the departure time of the travelers. The Bayesian multinomial logit regression was employed to explore the relationship between the travel mode choice and weather characteristics. The results showed that temperature, relative humidity, rainfall, wind, air quality index, and visibility had significant effects on the travel mode selection of travelers, and the addition of these variables could improve the model's predictive performance. The research results can provide a scientific decision basis for traveler flow transfer and the prediction of traffic modes choice due to the effects of climate change.

## 1. Introduction

High-speed rail (HSR) stations, airports, and other urban external transport hubs are important symbols of urban modernization and prosperity, and they greatly improve the efficiency of transportation. By the end of 2019, in China, the railway mileage reached 139,000 kilometers (35,000 kilometers are HSR), the highway mileage reached 143,000 kilometers, and there were 238 domestic transport airports (excluding Hong Kong, Macao, and Taiwan), including 39 airports with an annual traveler throughput of more than 10 million. These transportation infrastructures facilitate intercity communication and socioeconomic development. The travel modes of intercity traffic mainly include airplanes, HSR, conventional trains (termed as train), and express buses. The exploration of the factors influencing the choice of intercity travel mode is very important for the formulation of traffic demand management strategies.

To date, the individual characteristics [1–4], accessibility to transportation hubs [3–8], travel demand characteristics [2, 9], and travel mode characteristics [1, 2, 4, 5, 9] were found to have significant impacts on the intercity travel mode choice. Although some studies have explored the effect of weather on passengers' traffic mode choice in cities [10–14] and a few scholars have focused on the possible effects of weather characteristics on intercity transportation in the Netherlands, USA, and Spain [12, 13, 15–17]; the impact of weather on travelers' intercity mode choices has been ignored, especially in the case of Chinese cities.

This study aimed to explore the potential influence of weather conditions on the choice of intercity travel modes using a comprehensive dataset collected in Xi'an, China, in March 2019. The individual characteristics of travelers and revealed preference (RP) survey data of travelers' spring intercity travel activity were collected, and they were matched with the weather characteristics at the departure times of the travelers. The Bayesian multinomial logit (BMNL) regression was employed to analyze the relationships between the travel mode choice and the individual characteristics of travelers, intercity travel characteristics, and weather characteristics after correlation analysis and multicollinearity diagnosis of the independent variables. The study examines the possible influences of temperature, humidity, wind power, rainfall, air quality index, and visibility on travelers' intercity travel modes. It is expected to provide theoretical support and a decision-making basis for transportation planning, demand forecasting, and emergency management strategy formulation of integrated transportation networks due to climate change.

The rest of the paper is organized as follows: Section 2 reviews the impact of weather events on the choice of travel modes.  Section 3 describes the experiments, including survey subjects, questionnaire design, field investigations, and data characteristics.  Section 4 presents the methodology, including correlation analysis, multicollinearity diagnosis, and the structure, evaluation, and interpretation of the Bayesian multinomial logit model.  Section 5 presents the results of the study.  Section 6 summarizes the main findings, application value, and limitations of this study.

## 2. Literature Review

Previous studies have revealed the impact of weather conditions on the choice of urban transportation modes, including the season [10–12, 18], humidity [10–15], temperature [11–17], wind speed [10, 13–17], snow [10, 11, 16, 17], fog [10, 16], rain [15–17], the air quality index (AQI) [14], and extreme weather [18, 19]. For example, Böcker et al. [12] found car use seemed to be less attractive in spring, and travel by walking and cycling was less common in winter than in spring during 2004–2009 in the Randstad Holland. Chen and Wang [10] analyzed the on-time performance (OTP) records of aviation and HSR services from October 2016 to September 2017, revealing that the OTP of aviation is often significantly lower in summer, further confirming that the OTP of aviation is more susceptible to severe weather, such as heavy rainfall and thunderstorms.

Scholars have investigated the relationship between weather and travel choices by exploring various impacts of weather parameters, particularly precipitation and temperature [12]. Li et al. [11] reported that precipitation-related events were negatively related to daily ridership fluctuations at both levels of the single metro line and the metro network, using the data of weather and ridership in Nanjing from 2011 to 2014. Reference [14] found that walking was seldom affected by humidity according to the Beijing School Commute Survey during 2014–2015. In contrast, the share of the bicycle mode decreased greatly with the increase in humidity; the same results were obtained by Böcker et al. [12]. Chen and Wang [10] revealed that the precipitation in Beijing was negatively related to the change of the HSR's OTP, showing that precipitation increased by 1%, while HSR's OTP decreased by 0.019%.

For temperature, Hagenauer and Helbich [13] found that temperature was particularly important to predict bicycle and public transportation trips and generally more important than the precipitation or wind speed. However, Li et al. [11] reported that, compared with temperature-related events, precipitation-related events produced more significant traveler fluctuations, and temperature-related conditions could slightly reduce the daily metro traveler volume in Nanjing. Furthermore, it was suggested that the increase in temperature led to an increase in the number of trips using the ridership transit data in Gipuzkoa, Spain [15]. Böcker et al. [17] revealed that factors, such as low temperatures and, to some extent, rainfall and wind speed, could reduce the possibility of choosing cycling and outdoor leisure destinations in the part of study regions. The study of Ma et al. [14] showed that the increase of the highest temperature could reduce the attractiveness of walking and public transport. Cycling was the most affected by temperature, compared with walking, public transport, and car travel, and its market share was predicted to increase by 14.7% for a 4°C increase in the highest temperature.

As for wind, Ma et al. [14] revealed that an increase in the wind speed would lead to a decrease in walking, cycling, and use of public transport and an increase in car use. What is more, public transport was also not popular on windy days. Arana et al. [15] reported that the wind can produce a greater effect on Saturdays than on Sundays on the number of trips. Furthermore, Böcker et al. [17] found in Norway that wind would increase the combining of trips, resulting in more efficient trip chains, which may reduce weather exposure.

Recently, some scholars have found that rain and snow also affected the travel mode choice. Li et al. [11] showed that snowfall and large temperature deviations in winter lead to the drastic change in ridership. Singhal et al. [16] found that, in New York, heavy snow over midday weekdays may lead to an increase in ridership, while the heavy snow over midday and afternoon weekends may lead to a decrease in ridership. Furthermore, Chen and Wang [10] revealed that the negative influence of snowfall on HSR's OTP seemed to be more severe compared with other weather types. For example, the snowfall in Jinan reduced the HSR's OTP by 2.4%. Böcker et al. [17] found that travelers took short trips to reduce their exposure to snowfall in Stavanger and Utrecht. However, in Oslo and Stockholm, the effect of snow was insignificant, possibly because their citizens were more familiar with and resistant to snowfall. As for rain, Singhal et al. [16] suggested that rain had an impact on all periods on weekends, but midday and afternoon ridership were more significantly influenced than morning ridership. As for weekdays, compared with midday ridership, the rain had a greater impact on afternoon ridership. Arana et al. [15] concluded that if the wind and temperature were constant, adding one liter of rain per square meter would cause a decrease of 163 trips on Saturday and 104 trips on Sunday.

Several studies have revealed that other weather conditions have great influence on the choice of transportation mode. Weather conditions, such as sky conditions, wind speed, maximum temperature, humidity, air quality index (AQI), and their interactions, were found to be significantly associated with students' choice of commuting mode [14]. Ma et al. [14] reported that the change of air quality index from good to bad would lead to the decrease of the average probabilities of walking, cycling, and taking public transport by 3.4%, 5.9%, and 6.0%, respectively, while the probability of using cars increased by 14.7%. Ma et al. [14] also found that the change of sky conditions from good to bad would lead to decreases in the probabilities of walking, cycling, and taking public transport by 2.3%, 21.5%, and 2.1%, respectively. In addition, the number of students using car increased by 18.1%. Hyland et al. [18] used the survey data of Chicago travelers by Standard & Poor's to show that most respondents were less likely to choose cars to travel in bad weather than in good weather. Furthermore, Chen and Wang [10] concluded that the OTP of HSR in southeast coastal areas was more likely to be affected by rainstorms and thunderstorms than other weather conditions, while snowstorms seemed to be more destructive to HSR in the central-eastern and northern regions. Böcker et al. [17] revealed that dark skies (even at night) have negative impacts on the travel chain and the use of active transportation modes. Ton et al. [19] suggested that weather conditions had limited influence on cycling or walking by using census data from the Netherlands Mobility Panel.

The most widely used models in the intercity travel mode choice affected by weather conditions are still based on the utility theory of discrete selection models, including the multinomial logit (MNL) model [12, 14], multinomial probit (MNP) model [14], mixed multinomial logit model [19], and panel mixed logit model [18]. Other models have also been used, such as machine learning [13], moving average method [11], regression analysis [10, 15, 16], agent-based model [20, 21], and structural equation models (SEM) [17].  Table 1 presents a literature summary on the travel mode choice. Existing models typically used maximum likelihood estimation as a parameter estimation method [12, 14, 18, 19, 22]. The discrete choice modeling technology brings the development to the Bayesian parameter estimation method in the traffic safety field [23–25]. The Bayesian method has been shown to be able to better integrate implicit sample information, obtain parameter estimates with good statistical performances, and improve the efficiency of the model estimation [24, 25].

It is evident from previous studies that the research on the influence of weather on the travel mode choice is limited to urban transportation. Studies evaluating the effects of weather conditions on the intercity mode choice are rare. Moreover, the influence of weather conditions on the intercity mode choice varies with country, region, or even city. Therefore, this study analyzed the impact of weather on the intercity mode choice (i.e., airplane, HSR, train, and express bus) in Xi'an, China. This study would provide a more effective basis for the demand management of intercity transportation modes and the formulation of green development policies in the context of climate change.

## 3. Data Collection

### 3.1. Background Information

This study focused on the travelers traveling to and from Xi'an. Xi'an is an ancient central city in northwest China, with famous scenic attractions, such as the Qin Shi Huang Mausoleum, Bell Tower and Drum Tower, and Tang Paradise. Xi'an has a warm, temperate, semihumid mainland monsoon climate with four distinct seasons. March is the month when migrant workers go out to work and students return to school. Since March is a month between winter and spring in Xi'an, the temperature fluctuates, and the highest temperature can sometimes reach more than 20°, while the lowest temperature is only about 0°C. Furthermore, haze still exists to a large extent due to heating provided by the government from November 15 to March 15 in the previous year, the air visibility is relatively low, and there are more cloudy and rainy days, which has a potential impact on the travelers' intercity mode choice. In addition, from 2010 to 2018, the tourism revenue in Xi'an grew by about 15% annually. With the large-scale construction of high-speed railway lines, stations, and other infrastructure, the ways to meet the travel needs of tourists are becoming more and more diversified. Among all modes of transportation, express buses, HSRs, trains, and airplanes are often used by travelers.

### 3.2. Questionnaire Design

The questionnaire was designed to include three parts: (1) the individual attributes of the travelers, including gender, age, occupation, monthly income, and car ownership; (2) the travel attributes of the travelers, including the starting time for the carrier, origin city, destination city, the identification number of flight, train, HSR, or express bus, and travel purpose; (3) the travel-mode-related characteristics, including the access mode, access time, access cost, intercity travel mode, intercity travel cost, departure mode, departure time, and departure cost.

### 3.3. Field Investigations

This study was conducted through field investigations. The field investigations were conducted by eight well-trained undergraduate students who surveyed the Xi'an Xianyang airport, HSR station, railway station, and expressway traveler station from March 1 to 20, 2019. We applied the random sampling technique to this revealed preference survey [26, 27]. The investigators were instructed to randomly select one in every five travelers in their sampling area regardless of sex, age, or other factors [9]. The respondents were first told about the purpose of the survey and guaranteed that their answers would be anonymous. Then they were invited to participate in the survey. During the investigation, the investigator helps the respondents to understand the questions in the questionnaire.

### 3.4. Data Collation and Description

A total of 2200 original questionnaires were obtained through field investigations. During the data quality check, the data were excluded for the following reasons: (1) incomplete key information, (2) neither its origin nor its destination is Xi'an, or (3) the questionnaire having missing or incorrect data. Overall, there were 2028 valid samples. In addition, according to the origin and destination cities of the trip and the identification number of the chosen transportation mode, the intercity distance and travel time could be measured by using the Baidu map and the transportation schedules [9]. Based on the starting time for the chosen transportation mode, the weather information was obtained for the hour at which the carrier started. The travelers' travel activity data were matched with the weather condition data. The wind power and the AQI index were obtained from the weather forecast network (http://tianqi.2345.com/wea_history/57036.htm). The temperature, humidity, rainfall, and visibility were obtained from the national meteorological data-sharing platform (http://tianqi.2345.com/wea_history/57036.htm).

The basic statistics of the data were analyzed. The descriptions of the categorical variables are presented in Table 2, and the descriptions of the continuous variables are presented in Table 3.

## 4. Methodology

The BMNL was used for modeling. The traditional logit model is used to obtain the estimated parameters based on the maximum likelihood function, which is divided into fixed utility and random utility, where the random utility obeys a Gumbel distribution. Compared with the traditional discrete choice model based on probability, Bayesian inference can handle complex models and obtain better accuracy [23–25, 28–30]. Therefore, the Bayesian multinomial logit regression was used for parameter estimation.

This section first introduces the correlation analysis and multicollinearity test for the selection of independent variables. The BMNL model, odds ratio (OR) technique, and deviation information criterion were then introduced for parameter estimation, assessing the effect of significant factors, as well as model comparison, respectively.

### 4.1. Correlation Analysis of Independent Variables

The Pearson correlation coefficient is employed to measure the correlation between two variables. The Pearson correlation coefficient between two variables *P* and *Q* is defined as the quotient of the covariance of the two variables and the product of the standard deviation of the two variables as follows [31]:

(1) $$\begin{array}{c} \theta =\frac{\sum_{i=1}^{N}\left(P_{i}-\bar{P}\right)\left(Q_{i}-\bar{Q}\right)}{\sqrt{\sum_{i=1}^{N}{\left(P_{i}-\bar{P}\right)}^{2}}\sqrt{\sum_{i=1}^{n}{\left(Q_{i}-\bar{Q}\right)}^{2}}}. \end{array}$$

When the value of |*θ*| is closer to 1, it indicates a higher correlation between the two variables. Furthermore, the Pearson correlation coefficient is symmetric.  Table 4 shows the corresponding correlation degree of |*θ*|.

### 4.2. Multicollinearity Test

Multicollinearity refers to the distortion of the model estimate due to a high correlation between independent variables in the model [32, 33]. The variance inflation factor (VIF) was applied to measure the multicollinearity between independent variables. The specific formula of VIF for variable *x*_*k*_ is defined as follows:

(2) $$\begin{array}{c} {\text{VIF}}_{k}=\frac{1}{1-R_{k}^{2}}x_{k}, \end{array}$$

where *R*_*k*_^2^ represents the determination coefficient obtained by regression with *x*_*k*_ as the dependent variable and the other variables as independent variables. A larger VIF corresponds to greater collinearity. If the VIF is greater than 5, there is a significant multicollinearity between this variable and other variables [32].

### 4.3. Bayesian Multinomial Logit Model

The BMNL model was established to determine how various factors influence a traveler's intercity mode choice [34, 35]. The specific formula can be expressed as follows [9, 36]:

(3) $$\begin{array}{c} P\left(Y_{i}=j\right)=\frac{\exp\left(\delta_{0j}+\delta_{1j}x_{1i}+\delta_{2j}x_{2i}+\cdots +\delta_{kj}x_{ki}\right)}{\sum_{m=1}^{J}\left(\delta_{0m}+\delta_{1m}x_{1i}+\delta_{2m}x_{2i}+\cdots +\delta_{km}x_{ki}\right)}, \end{array}$$

where *Y*_*i*_=*j* corresponds to sample *i* selecting transportation mode *j*, *x*_*ki*_ indicates the value of variable *k* for sample *i*, *δ*_*kj*_ is the coefficient of variable *k* for transportation mode *j*, and *J* is the total number of transportation modes. The likelihood function of BMNL can be expressed as follows:

(4) $$\begin{array}{c} f\left(Y|\delta \right)=\prod_{i=1}^{N}\prod_{j=1}^{J}\left[d_{ij}\times P\left(Y_{i}=j\right)\right]=\prod_{i=1}^{N}\prod_{j=1}^{J}\left[d_{ij}\times \frac{\exp\left(\delta_{0j}+\delta_{1j}x_{1i}+\delta_{2j}x_{2i}+\cdots +\delta_{kj}x_{ki}\right)}{\sum_{m=1}^{J}\delta_{0m}+\delta_{1m}x_{1i}+\delta_{2m}x_{2i}+\cdots +\delta_{km}x_{ki}}\right], \end{array}$$

where N is the sample size, *d*_*ij*_ is an indicator which equals 1 if the discrete outcome for sample *i* is *j* and 0 otherwise, and *δ*=[*δ*_0_, *δ*_1_, *δ*_2_,…,*δ*_*k*_]^*T*^ is the parameter vector.

A Bayesian inference approach based on Markov Chain Monte Carlo (MCMC) method was used to simulate the posterior distribution of *δ*. The estimates of the mean, standard deviation, and quartiles of the parameters of each explanatory variable can be determined by the posterior distribution provided by the Bayesian approach [23]. Based on the specification of the Bayes theorem, the posterior distribution of parameters can be estimated using the following function:

(5) $$\begin{array}{c} f\left(\delta |Y\right)=\frac{f\left(Y,\delta \right)}{f\left(Y\right)}=\frac{f\left(Y|\delta \right)\pi \left(\delta \right)}{{}^{\int f\left(Y|\delta \right)\pi \left(\delta \right)\text{d}\delta }}\propto f\left(Y|\delta \right)\pi \left(\delta \right), \end{array}$$

where *f*(*δ| ***Y**) denotes the posterior joint distribution of parameter *δ* conditional on dataset *Y*.  *f*(**Y**,  *δ*) represents the joint probability distribution of dataset **Y** and model parameter *δ*. *f*(*δ| ***Y**) is the likelihood conditional function based on parameter *δ*, specified by equation (4). Function *π*(*δ*) is the prior distribution of parameter *δ* [9]. Due to the lack of information on the random parameters, the following noninformative prior distributions for parameter *δ* were used:

(6) $$\begin{array}{c} \delta ∼N\left(0_{k},10^{6}I_{k}\right), \end{array}$$

where 0_*k*_ is a vector of zeros and **I**_*k*_ is a *k* × *k* identity matrix.

The posterior joint distribution *f*(*δ| ***Y**) can be derived as follows:

(7) $$\begin{array}{c} f\left(\delta |Y\right)\propto f\left(Y|\delta \right)=\prod_{i=1}^{N}\prod_{j=1}^{J}\left[d_{ij}\times \frac{\exp\left(\delta_{0j}+\delta_{1j}x_{1i}+\delta_{2j}x_{2i}+\cdots +\delta_{kj}x_{ki}\right)}{\sum_{m=1}^{J}\delta_{0m}+\delta_{1m}x_{1i}+\delta_{2m}x_{2i}+\cdots +\delta_{km}x_{ki}}\right]\times \prod_{i=1}^{N}\prod_{j=1}^{J}\left[\frac{1}{\sqrt{2\pi }10^{3}}\exp\left(-\frac{1}{2}\frac{{\left(\delta_{kj}\right)}^{2}}{10^{6}}\right)\right],\\ \propto \;\exp\left\{\sum_{i=1}^{N}\sum_{j=1}^{J}\left[d_{ij}\times \frac{\exp\left(\delta_{0j}+\delta_{1j}x_{1i}+\delta_{2j}x_{2i}+\cdots +\delta_{kj}x_{ki}\right)}{\sum_{m=1}^{J}\delta_{0m}+\delta_{1m}x_{1i}+\delta_{2m}x_{2i}+\cdots +\delta_{km}x_{ki}}\right]\right.\left.-\sum_{i=1}^{N}\sum_{j=1}^{J}\left[\frac{1}{2}\frac{{\left(\delta_{kj}\right)}^{2}}{10^{6}}\right]\right\}. \end{array}$$

To generate realizations from the posterior joint distribution *f*(*δ| ***Y**), the Metropolis-Hasting sampling approach sequentially draws parameters from equation (7). The inference can then be made based on the remaining draws after discarding the draws during the burn-in period.

### 4.4. Odds Ratio

The OR was applied to measure the influence of the explanatory variables. It represents the increase in the odds of the outcome if the value of the variable increased by one unit [9, 22, 37]. The OR of variable *x*_*k*_ corresponding to mode *j* can be calculated as

(8) $$\begin{array}{c} \text{OR}=\frac{\text{odds}\left(X,x_{kj}+1\right)}{\text{odds}\left(X,x_{kj}\right)}=\frac{\exp\left(X\delta \right)\times \;\exp\left(\delta_{kj}\right)}{\exp\left(X\delta \right)}=\exp\left(\delta_{kj}\right). \end{array}$$

### 4.5. Deviation Information Criterion

The deviation information criterion (DIC) was used to compare the fitting performance in the Bayesian model [38]. The formula is as follows [39]:

(9) $$\begin{array}{c} \text{DIC}=\bar{D}+S_{D},\\ \bar{D}=f_{\begin{array}{c} \left(\delta |Y\right) \end{array}}\left[-2f\left(Y|\delta \right)\right],\\ S_{D}=f_{\left(\delta |Y\right)}\left[-f\left(Y|\bar{\delta }\right)\right],\\ \bar{\delta }=f_{\left(\delta |Y\right)}, \end{array}$$

where *f*(*Y|δ*) is the likelihood function of the model, $\bar{\delta }$ is the posterior mean of *δ*, which can be written as $\bar{\delta }=f_{\left(\delta |Y\right)}$, and *f*_(*δ|Y*)_(*X*) is the mean of *X* under the posterior distribution of *π*(*δ|Y*). For model comparison, a lower DIC represents a higher model accuracy for parameter estimation and prediction.

## 5. Results

### 5.1. Selection of Independent Variables

The correlation analysis results are shown in Table 5. Gender, age, occupation, monthly income, car ownership, travel purpose, travel distance, intercity travel time, intercity travel cost, temperature, relative humidity, rainfall, wind power, AQI, and visibility are found to be correlated with the intercity travel mode choice. Second, the variables that are significantly related to the travel mode choice and do not cause bias estimates for other variables are selected to be kept in the model. Finally, sex, age, occupation, monthly income, travel purposes, travel distance, temperature, relative humidity, rainfall, wind speed, air quality, and visibility were included in the model. The collinearity diagnosis results are presented in Table 6, and no collinearity characteristics were evident.

### 5.2. Parameter Estimates

Table 7 presents the parameter estimation results using the BMNL model without the weather variables.  Table 8 shows the parameter estimate results from the BMNL model considering the weather variables. The mean and SD in Tables 7 and 8 represent the mean values and the standard deviation of the posterior distribution, respectively. 2.5% and 97.5% were the lower and the upper limits of the 95% confidence interval, respectively. If a parameter's confidence interval did not include 0, this factor was considered to be significantly associated with the choice of the traveler's travel mode. Only significant variables were kept in Tables 7 and 8.

### 5.3. Factor Analysis

As shown in Tables 7 and 8, the DIC values of the models without and with weather variables were 4530.322 and 4078.377, respectively. The small DIC of the model with the weather conditions indicated that the weather could enhance the predictive accuracy of the travel mode choice model. Therefore, the analysis of various variables in this study was based on the estimation of the parameters from the model considering the weather conditions.

#### 5.3.1. Gender

As shown in Table 7, gender was significantly correlated to airplane choice, and the mean of the variable was positive, showing that male travelers were more likely to choose airplane travel than female travelers. For the train and express bus, the negative mean of the gender indicated that male travelers were less likely to select these travel modes than female travelers. The OR of the gender for airplane travel was 1.1239, indicating that male travelers were 12.39% more likely to select airplanes than female travelers. For train and bus, the ORs were 0.5388 and 0.6393, respectively, indicating that male travelers were 46.12% and 36.07% less likely to select bus and train than female travelers, respectively.

#### 5.3.2. Age

Age was found to have a negative effect on the choice of airplane or express bus travel compared with HSR travel. Thus, older travelers were less likely to choose airplanes and express buses than HSR. Compared to HSRs, the ORs of the age for airplane and express bus travel were 0.9241 and 0.9150, respectively, indicating that each increase in 10 years of age will cause a 7.59% decrease in odds of selecting an airplane and an 8.85% decrease in odds of selecting an express bus. In addition, age had no significant effect on travelers' train choice. These results are similar to those of a previous study [9], indicating that older travelers prefer to choose HSR travel compared to express buses.

#### 5.3.3. Occupation

The negative correlation between students' choice of airplanes and express bus showed that students were more unlikely to select airplane and express bus travel than government or company employees. The ORs of the students for airplanes and express buses were 0.6004 and 0.6801, respectively, indicating that the odds of students choosing airplanes and express buses were reduced by 39.96% and 31.99%, respectively, compared with government or company employees. For trains, the mean of the students was positive, showing that students were more likely to choose train than government or company employees. The OR of the students for train travel was 1.4053, which indicated that the odds of students choosing train travel were 40.53% greater than those for government or company employees. This may result from a lack of personal financial resources, causing students to select a relatively cheap travel mode.

Compared with HSR, self-employment was positively associated with airplane choice, train, and express bus travel, indicating that self-employed travelers preferred to choose these travel modes than government or company employees. The ORs of self-employed travelers were 1.1777, 2.9946, and 3.2638 for airplane, train, and bus travel, respectively, corresponding to 17.77%, 199.46%, and 226.38% increased odds of choosing these modes, respectively, compared with government or company employees.

Farmers or people with other professions had negative correlations with the choice of airplanes, indicating that farmers or other employees were less likely to choose airplane travel. The OR of farmers or others was 0.7741, indicating that these people were 22.59% less likely to choose airplane travel than government or company employees. For train and express bus choice, the correlations with farmers or other professions were positive, indicating that more farmers or people in other professions preferred to select trains and express buses than government or company employees, with ORs of 2.2368 and 2.5130, respectively. This indicated that farmers or people in other professions were 123.68% and 151.30% more likely to choose train and express bus travel than government and company employees.

#### 5.3.4. Monthly Income

The correlation of monthly income was negative with the choice of the airplane, train, and express bus travel, indicating that a higher monthly income corresponded to a smaller probability of travelers choosing airplane, train, and express bus travel compared with HSR. The corresponding ORs of monthly income were 0.8485, 0.7531, and 0.6959, which indicated that, for every 1000 Yuan increase in monthly income, the odds of travelers choosing airplane, train, and express bus travel increased by 15.15%, 24.69%, and 30.41%, respectively.

#### 5.3.5. Travel Purpose

Compared with HSR, travel purpose (leisure travel versus mandatory travel) is insignificantly related to airplane choice. The positive sign of travel purpose with train and express bus choice indicated that more leisure travel travelers preferred to choose train and express bus travel than compulsory travel travelers. The ORs of travel purpose for railway and express bus travel were 1.5122 and 1.7364, respectively. This indicated that the odds of travelers traveling for leisure purposes choosing train and express bus travel were, respectively, 51.22% and 73.64% greater than those for mandatory travel.

#### 5.3.6. Travel Distance

For airplane travel, the positive correlation with the travel distance indicated that, for longer travel distances, travelers were inclined to select airplanes. Compared with HSR, the odds of choosing an airplane and train increased by 0.16% and 0.03%, respectively, for every 1 km increase of travel distance. The correlation of the travel distance with the express bus choice was negative, which indicated that a longer travel distance corresponded to a smaller probability of travelers choosing express bus travel. Compared with HSR, the odds of selecting an express bus decreased by 0.31% for every 1 km of travel distance.

#### 5.3.7. Temperature

The temperature was negatively correlated with the choice of the airplane and express bus travel, indicating that a higher temperature corresponded to a smaller probability of the travelers choosing airplane and express bus travel. The advantage ratios of the temperature were 0.7290 and 0.6062, respectively, which indicated that, for every 5°C increase in temperature, the odds of choosing airplane and express bus travel over HSR decreased by 27.1% and 39.38%, respectively. For train, the correlation with the temperature was positive, indicating that a higher temperature corresponded to a greater probability of travelers choosing train travel. The advantage ratio of the temperature was 1.1856, which indicated that, for every 5°C increase in temperature, the odds of choosing train travel over HSR increased by 18.56%.

#### 5.3.8. Relative Humidity

The negative influence of relative humidity on the choice of airplane, train, and express bus travel indicated that the greater the relative humidity was, the smaller the probability of travelers choosing these travel modes became. The advantage ratios of relative humidity were 0.9910, 0.9575, and 0.9809, which indicated that, for each percentage increase in the relative humidity, compared with HSR, the probability of choosing airplane, train, and express bus travel decreased by 0.9%, 4.25%, and 1.91%, respectively.

#### 5.3.9. Rainfall

For the choice of airplane and train travel, the impact of rainfall was negative, indicating that, with a greater amount of rainfall, the probabilities of travelers selecting these travel modes were smaller. Compared with HSR, the odds of choosing airplane and train travel were reduced by 16.04% and 10.53% for each 1 mm increase in rainfall. Compared with HSR, rainfall had no significant effect on express bus choice.

#### 5.3.10. Wind Power

Compared with HSR, wind power had no significant effect on choosing airplane travel. A possible reason for this is that Xi'an, China, is located in a warm, temperate, semihumid mainland monsoon climate, with less wind in spring and less impact on airplane and HSR delays. The mean of the wind power for train and express bus travel was negative, showing that the greater the wind power was, the smaller the odds of travelers choosing train and bus travel became. The ORs of wind were 0.7020 and 0.8330, respectively, which showed that, for each unit of wind increase, compared with HSR, the odds of choosing train and express bus travel were reduced by 29.8% and 16.7% respectively.

#### 5.3.11. Air Quality Index

For airplanes and trains, the positive impact of the AQI indicated that the better the AQI was, the greater the odds of travelers selecting these travel modes became. The AQI corresponded to ORs of 1.0054 and 1.0033, respectively, indicating that, compared with HSR, for an AQI increase of 1 *μ*g/m^3^, the odds of selecting airplane and train travel increased by 0.54% and 0.33%, respectively. The AQI mean value was negative for the express bus, showing that the better the AQI was, the smaller the odds of travelers selecting express bus travel became. The AQI for express bus travel corresponded to an OR of 0.99898, indicating that, compared with HSR, an increase in the AQI of 1 *μ*g/m^3^ decreased the odds of selecting express bus travel by 1.02%.

#### 5.3.12. Visibility

For airplane, train, and express bus travel, the positive sign of the visibility indicated that, with better visibility, the odds of travelers choosing airplane, train, and express bus travel were greater. The ORs of these modes were 1.003, 1.0001, and 1.0005, respectively, indicating that, compared with HSR, an increase of 1 m of visibility corresponded to increased odds of selecting airplane, train, and express bus travel of 0.03%, 0.01%, and 0.05%, respectively.

## 6. Discussion and Conclusions

This study investigated the travel activity data of travelers arriving in and leaving Xi'an, China, in March 2020 by airplane, HSR, train, and express bus, and the weather characteristics at the traveler departure time were matched with the travel activity data of the travelers. Based on the independent variable correlation analysis and multicollinearity test, the BMNL model was used to estimate the parameters. The effect of significant influencing factors was quantitatively evaluated by OR technology. The results can provide theoretical support and a decision basis for the planning and demand management of intercity transportation networks due to climate change. The specific research conclusions and application values are as follows.

In addition to the traditional individual attributes of travelers (gender, age, occupation, and monthly income) and travel demand attributes (travel purpose and travel distance), weather conditions (i.e., temperature, relative humidity, rainfall, AQI, and visibility) also had significant impacts on the intercity travel mode choice.

The results showed that, for every 5°C increase in temperature, the odds of choosing airplane and express bus travel over HSR will decrease by 27.1% and 39.38%, respectively, and the odds of choosing train travel will increase by 18.56%. This can provide a basis for future integrated traffic network planning. In the current global warming context, the increase in temperature will lead to travelers being more willing to travel by rail. China's railway, especially HSR, has adapted to the travel needs of travelers in the context of global warming. On the one hand, this conclusion fully validates China's development of HSR from the perspective of the environment. On the other hand, it also provides theoretical support for the development of HSRs in other countries in response to climate change.

The relative humidity negatively affected the travelers' airplane, train, and express bus choice compared with the HSR. The higher relative humidity causes travelers to feel wet; especially when the temperature is high, it will give the traveler a feeling of sultry heat, which significantly affects travel. Therefore, operators should improve the air quality inside the railway and express bus carriages and enhance the attractiveness of traffic modes.

The odds of choosing airplane and train travel will be reduced by 16.04% and 10.53% per 1 mm increase in rainfall, respectively. Rainfall has a great influence on intercity travel. When there is a large amount of rainfall, the delay of the airplane will increase greatly. It is necessary to guide travelers to other modes of transportation, such as HSR and train travel.

Wind power was negatively associated with the choice of conventional train and express bus. For each unit of wind increase, the odds of choosing train and express bus travel will be reduced by 29.8% and 16.7%, respectively. Wind power had little influence on the choice of intercity mode in this study. The main reason for this was that the data used in this study were from Xi'an, China, in spring, while the wind power in Xi'an, China, in spring is relatively small. When the wind power is large, it will generally affect the travel of various modes of transportation, especially airplane travel. Therefore, the traffic management department should reasonably establish contact with the meteorological department, the tourism department, and other relevant departments of the city. When the meteorological department predicts the existence of severe weather, such as strong wind and heavy rain, the city manager should publish the information in time and take corresponding measures to reduce unnecessary, nonmandatory travel, especially for coastal areas prone to typhoons and rainstorms.

The AQI had a significant positive effect on airplane and train travel. The odds of travelers selecting these modes will increase by, respectively, 0.54% and 0.33% for every 1 *μ*g/m^3^ increase in the AQI. The AQI had a significant negative effect on express bus travel, with a 1.02% decrease in odds of selecting this mode for every 1 *μ*g/m^3^ increase of the AQI.

Visibility had a significant positive impact on airplane, train, and express bus travel. For each 1 mm increase in visibility, the probability of travelers selecting airplane, train, and express bus travel will increase by 0.3%, 0.01%, and 0.05%, respectively. AQI and visibility mainly affect the intercity travel environment and driving visibility. With the industrialization in China, urban air quality has continually declined, which causes haze. This significantly affects the health of travelers and travel comfort. As reported by [40], public awareness of haze has an important influence on domestic travel in China. Therefore, for tourist cities such as Xi'an, it is important to improve the environment on which humans depend.

There were still some limitations in this study. First, only the travel activity and weather data of travelers entering and leaving Xi'an, in March, were examined. The seasonal variation of weather conditions in this one city may have affected the choice of travel mode. Therefore, in future research, the influence of seasonal changes on the intercity travel mode should be considered, and the impact of the weather on the selection of traveler intercity travel modes in different seasons should be explored. Furthermore, Xi'an is located in the northwest of China. It has a warm, temperate, semihumid Mainland monsoon climate, which has significantly different urban climate characteristics compared to the southeast coast of China and northeast China. In future research, cities with different climatic characteristics can be selected to explore the influence of weather on traveler intercity travel mode choice.

In addition, more advanced models, such as the Bayesian mixed effect model, can also be used to further reveal the unobservable heterogeneity of weather on the choice of traveler intercity modes, and other machine learning models, such as C 5.0 and random tree, could be applied to this study to determine the relative importance of various weather variables. Finally, the sample number of different traffic modes in this study is unbalanced to a certain extent, and whether the data imbalance will have a significant impact on the fitting and prediction performance of the model needs to be explored in subsequent studies.

## Figures and Tables

**Table 1:** Summary of previous literature.

Authors and year	Data source	Travel mode	Weather condition	Modeling approach	Main findings
Hagenauer and helbich [13]	The Dutch National Travel Survey (NTS), data from 2010 to 2012	Walking, bike, car, public transport	Precipitation, temperature, wind speed	Machine learning, multinomial logit (MNL), naive Bayes (NB), support vector machine (SVM), and artificial neural network (ANN)	Temperature is particularly important in predicting bicycle and public transportation trips, and it is often more important than precipitation or wind speed in determining transportation mode choices
Li et al. [11]	The weather and ridership data in Nanjing from 2011 to 2014	Metro	Precipitation, temperature, seasonality	Moving average method, analysis of variance (ANOVA) models	Compared with temperature-related events, precipitation-related events produce more significant ridership fluctuations. The temperature-related events only slightly decrease metro daily ridership in Nanjing.
Böcker et al. [12]	Data from all seasons from 2004 to 2009 in Randstad, Netherlands	Walking, cycling, car, public transport	Precipitation, temperature	Multinomial logit model	The use of car seems to be less attractive in spring. However, positive effects on walking and especially cycling seem to be less pronounced than in winter.
Ton et al. [19]	Census data from the Netherlands Mobility Panel (MPN)	Car, public transport, bicycle, walking	Season and weather characteristics	Mixed multinomial logit	The weather has a limited impact on active mode choice
Ma et al. [14]	The Beijing school commute survey data from 2014 to 2015	Walking, bicycle, public transport, car	Sky conditions, wind speed, highest temperature, lowest temperature, air quality index, humidity	Multinomial probit (MNP) and multinomial logit (MNL) models	When the air quality is very bad, students are more inclined to take public transportation than cars. It may be that Beijing's special urban traffic regulations limit family car ownership and car use.
Singhal et al. [16]	New York subway ridership data for 2010-2011	Bus station, rail station	Temperature, wind, rain, snow, fog	Ordinary least squares (OLS) regression models, separate models, backward substitution method	The rain had a negative effect on subway ridership at all hours of the weekend. Midday and afternoon subway ridership is more severely affected than afternoon traffic.
Arana et al. [15]	Transit ridership data in Gipuzkoa, Spain	Bus	Temperature, relative air humidity, rain, wind	Multiple linear regression	Wind and rain could decrease the number of trips, while the rise of temperature could make the number of trips increase.
Chen and Wang [10]	The on-time performance records of HSR and air services from October 2016 to September 2017	HSR, aviation	Precipitation, fog, thunderstorm, wind, snow, season	Regression analysis	Compared with other weather types, the negative impact of snowfall on on-time performance of HSR is more serious
Hyland et al. [18]	Data from stated-preference (SP) survey of travelers in Chicago	Car, traditional transit, flexible transit	Good weather, bad weather	Panel mixed logit	Millennials are less likely to choose a car in winter than in summer. However, seasonality has little impact on nonmillennials' car choices.
Böckere et al. [17]	The national travel data in Norway (2013-2014), Sweden (2011), and Netherlands (2010–2012)	Walking, bicycle, public transport, car	Nighttime, darkness, air temp, wind speed, rainfall, snowfall	Structural equation modeling (SEM)	The dry and warm weather in Oslo and calm and dry weather in Stavanger increase the visitation of outdoor leisure destinations relative to work trips, but none of these effects were found in the non-Norwegian regions

**Table 2:** Description of categorical variables.

Variables	Category	Code	Frequency	Proportion
Dependent variable				
Mode choice	Airplane	1	460	22.68%
	HSR	2	774	38.17%
	Train	3	496	24.46%
	Express bus	4	298	14.69%
Independent variables				
Sex	Female	0	1026	50.59%
	Male	1	1002	49.41%
Age	0−19 years	1	175	8.63%
	20−29 years	2	937	46.20%
	30−39 years	3	399	19.67%
	40−49 years	4	297	14.64%
	50−59 years	5	202	9.96%
	Above 60 years	6	18	0.89%
Occupation	Government or company employees	1	868	42.80%
	Students	2	624	30.77%
	Self-employed	3	167	8.23%
	Farmers and others	4	369	18.20%
Monthly income	0−3000 Yuan	1	741	36.57%
	3000−4000 Yuan	2	565	27.89%
	4000−5000 Yuan	4	260	12.83%
	5000−6000 Yuan	5	207	10.22%
	≥6000 Yuan	6	253	12.49%
Car ownership	Yes	0	977	48.18%
	No	1	1,051	51.82%
Temperature	≥25°C	1	96	4.73%
	15−25°C	2	1127	55.57%
	10−15°C	3	547	26.97%
	5−10°C	4	211	10.40%
	0−5°C	5	47	2.32%
Travel purpose	Mandatory travel	0	1032	0.5089
	Leisure travel	1	996	0.4911

**Table 3:** Description of continuous variables.

Variables	Unit	Mean	SD	Minimum	Maximum
Relative humidity	%	40.170	21.976	0	90
Rainfall	mm	0.525	2.346	0	54
Wind power	Scale	2.313	1.010	0	8
Air quality index	—	101.324	54.600	5	387
Visibility	m	5528.418	858.161	216	8200
Travel distance	km	894.041	646.304	0	8748

**Table 4:** Relationship between |*θ*| and correlation degree [31].

Range of |*θ*|	Correlation degree
0.00–0.19	Very low correlation
0.20–0.39	Low correlation
0.40–0.69	Moderate correlation
0.70–0.89	Highly correlation
0.90–1.00	Extremely high correlation

**Table 5:** The correlation analysis results.

Variables	Intercity mode	Gender	Age	Occupation	Monthly income	Car ownership	Travel purpose	Travel distance	Temperature	Relative humidity	Rainfall	Wind power	Air quality index	Visibility
Intercity mode	1													
Gender	−0.1401^*∗*^	1												
Age	−0.0252^*∗*^	0.0077	1											
Occupation	0.2244^*∗*^	−0.0484^*∗*^	−0.065^*∗*^	1										
Monthly income	0.1515^*∗*^	−0.0646^*∗*^	−0.287^*∗*^	−0.1591^*∗*^	1									
Car ownership	0.1236^*∗*^	−0.0566^*∗*^	0.0491^*∗*^	−0.0766^*∗*^	0.1463^*∗*^	1								
Travel purpose	0.1411^*∗*^	0.0406	0.0044	0.1161^*∗*^	−0.0819^*∗*^	−0.0634^*∗*^	1							
Travel distance	−0.4378^*∗*^	0.029	0.0084	−0.0968^*∗*^	0.1444^*∗*^	0.0747^*∗*^	−0.0921^*∗*^	1						
Temperature	−0.0166	0.0111	−0.0749^*∗*^	−0.0441^*∗*^	−0.0289	0.0563^*∗*^	−0.0252	0.014	1					
Relative humidity	−0.3046^*∗*^	0.0697^*∗*^	−0.0475^*∗*^	−0.1906^*∗*^	0.0042	−0.0072	−0.0269	0.1457	0.2879	1				
Rainfall	−0.0784^*∗*^	0.0289	−0.0494^*∗*^	−0.1213^*∗*^	0.0754^*∗*^	0.1297^*∗*^	−0.0515^*∗*^	0.1011^*∗*^	0.2732^*∗*^	0.3104^*∗*^	1			
Wind power	−0.1282^*∗*^	0.0679^*∗*^	0.0407	−0.034	−0.0533^*∗*^	0.0529^*∗*^	-0.0319	0.0356	−0.1096^*∗*^	0.1002^*∗*^	−0.0242	1		
Air quality index	−0.0732^*∗*^	0.0291	0.0285	0.0263	−0.1849^*∗*^	−0.0441^*∗*^	0.0064^*∗*^	−0.0284	0.0845^*∗*^	0.0735^*∗*^	−0.0939^*∗*^	0.1674^*∗*^	1	
Visibility	0.0856^*∗*^	−0.0138	0.031	0.0152	0.0575^*∗*^	0.1598^*∗*^	-0.0328	−0.0145	0.0205	−0.2828^*∗*^	−0.0745^*∗*^	−0.0854^*∗*^	0.2217^*∗*^	1

^*∗*^ indicates that the variable was significant at 95% confidence level.

**Table 6:** The multicollinear diagnosis results.

Variables	VIF
Gender	1.03
Age	1.48
Occupation	1.10
Monthly income	1.71
Travel purpose	1.04
Travel distance	1.06
Temperature	1.20
Relative humidity	1.36
Rainfall	1.29
Wind speed	1.08
Air quality index	1.15
Visibility	1.16

**Table 7:** Parameter estimate results from Bayesian multinomial logit method without weather variables.

Variables	Airplane					Train					Express bus				
	Mean	SD	2.5%	97.5%	OR	Mean	SD	2.5%	97.5%	OR	Mean	SD	2.5%	97.5%	OR
Gender	——	——	——	——	——	−0.7139	0.1012	−0.9121	−0.5221	0.4897	−0.5321	0.1683	−0.8489	−0.1997	0.5874
Age	——	——	——	——	——	——	——	——	——	——	−0.1699	0.0492	−0.2648	−0.0751	0.8438
Occupation															
*Students versus government or company employees*	−0.4038	0.1720	−0.7145	−0.0420	0.6678	0.2432	0.1217	0.0032	0.4801	1.2753	−0.6155	0.2284	−1.0140	−0.1317	0.5404
*Self-employed versus government or company employees*	0.2939	0.1040	0.0802	0.4867	1.3417	1.6053	0.1571	1.2878	1.9094	4.9795	1.4421	0.2570	1.0158	2.0139	4.2297
*Farmers or others versus government or company employees*	——	——	——	——	——	1.2218	0.1148	1.0110	1.4667	3.3932	1.0534	0.1916	0.7109	1.4568	2.8674
Monthly income	−0.1840	0.0388	−0.2539	−0.1077	0.8319	−0.2980	0.0374	−0.3719	−0.2232	0.7423	−0.2441	0.0506	−0.3476	−0.1464	0.7834
Travel purpose															
*Mandatory travel versus leisure travel*	——	——	——	——	——	0.3401	0.0425	0.2573	0.4231	1.4050	0.6226	0.1428	0.3469	0.9013	1.8637
Travel distance	0.0013	0.0001	0.0011	0.0016	1.0013	——	——	——	——	——	−0.0030	0.0002	−0.0034	−0.0026	0.9970
Constant	−1.4270	0.2724	−1.9575	−0.8826	0.2400	−0.0112	0.1060	−0.2166	0.1989	0.9889	1.5659	0.2375	1.0559	1.9666	4.7872
DIC	4530.322														

**Table 8:** Parameters estimate results from Bayesian multinomial logit method with weather variables.

Variables	Airplane					Train					Express bus				
	Mean	SD	2.5%	97.5%	OR	Mean	SD	2.5%	97.5%	OR	Mean	SD	2.5%	97.5%	OR
Gender	0.1168	0.0495	0.0167	0.2133	1.1239	−0.6183	0.0192	−0.6567	−0.5872	0.5388	−0.4473	0.0184	−0.4772	−0.4116	0.6393
Age	−0.0790	0.0340	−0.1454	−0.0055	0.9241	——	——	——	——	——	−0.0889	0.0330	−0.1487	−0.0213	0.9150
Occupation															
*Students versus government or company employees*	−0.5102	0.0671	−0.6275	−0.4079	0.6004	0.3403	0.0368	0.2698	0.3951	1.4053	−0.3856	0.0212	−0.4206	−0.3514	0.6801
*Self-employed versus government or company employees*	0.1635	0.0292	0.1070	0.2212	1.1777	1.0968	0.0269	1.0484	1.1502	2.9946	1.1829	0.0182	1.1500	1.2198	3.2638
*Farmers or others versus government or company employees*	−0.2561	0.0361	−0.3227	−0.1848	0.7741	0.8050	0.0194	0.7667	0.8416	2.2368	0.9215	0.0230	0.8814	0.9715	2.5130
Monthly income	−0.1642	0.0214	−0.2030	−0.1197	0.8485	−0.2836	0.0116	−0.3062	−0.2623	0.7531	−0.3626	0.0289	−0.4196	−0.3122	0.6959
Travel purpose															
*Mandatory travel versus leisure travel*	——	——	——	——	——	0.4135	0.0435	0.3290	0.4791	1.5122	0.5518	0.0316	0.4843	0.6060	1.7364
Travel distance	0.0016	0.0001	0.0014	0.0018	1.0016	0.0003	0.0001	0.0001	0.0006	1.0003	−0.0031	0.0002	−0.0036	−0.0027	0.9969
Temperature	−0.3161	0.0193	−0.3543	−0.2777	0.7290	0.1703	0.0093	0.1534	0.1872	1.1856	−0.5005	0.0083	−0.5172	−0.4846	0.6062
Relative humidity	−0.0090	0.0032	−0.0152	−0.0026	0.9910	−0.0434	0.0034	−0.0500	−0.0367	0.9575	−0.0193	0.0037	−0.0267	−0.0123	0.9809
Rainfall	−0.1749	0.0251	−0.2147	−0.1299	0.8396	−0.1113	0.0338	−0.1753	−0.0616	0.8947	——	——	——	——	——
Wind power	——	——	——	——	——	−0.3538	0.0444	−0.4427	−0.2700	0.7020	−0.1828	0.0374	−0.2493	−0.1205	0.8330
Air quality index	0.0054	0.0011	0.0033	0.0074	1.0054	0.0033	0.0011	0.0011	0.0056	1.0033	−0.0102	0.0020	−0.0142	−0.0063	0.9898
Visibility	0.0003	0.0000	0.0002	0.0004	1.0003	0.0000	0.0000	0.0000	0.0001	1.0001	0.0005	0.0001	0.0004	0.0006	1.0005
Constant	−2.4953	0.0527	−2.5899	−2.3824	0.0825	1.3740	0.0451	1.3047	1.4685	3.9510	2.0775	0.0314	2.0248	2.1284	7.9849
DIC	4078.377														

## Data Availability

The data used to support the findings of this study are available from the corresponding author upon request.
